The article "An Empirical Study on the Relationship between New Energy Vehicle' Export Sophistication and Industrial Structure Upgrading in China" was retracted in 2023. Reasons: signs of a paper mill; compromised peer review; unreliable results or conclusions.

# An Empirical Study on the Relationship between New Energy Vehicle' Export Sophistication and Industrial Structure Upgrading in China

**DOI:** 10.1155/2022/8914898

**Published:** 2022-09-07

**Authors:** Xuwen Cao, Rajah Rasiah, Fumitaka Furuoka

**Affiliations:** Asia Europe Institute, University of Malaya, Kuala Lumpur, Malaysia

## Abstract

Following decades of reducing greenhouse gas emissions in the transportation industry, most car companies will stop producing petrol cars and promote the development of new energy vehicles in the near future, even in China. This study is based on energy vehicle exports using China's 31 provinces' panel data from 2010 to 2020. Considering that China mainly engages in processing trade, this study analyzes the domestic energy vehicle's export sophistication after deleting intermediate goods, measuring the relationship between export sophistication and industrial upgrading with static and dynamic panel models. Then, heterogeneity tests were deployed to examine the domestic export sophistication of three major economic belts partition. The results revealed that improving export sophistication is conducive to realizing China's industrial upgrading. China's new energy vehicles industry is positively affected by export sophistication, R&D, foreign direct investment, average GDP growth rate, market factors, and human resources over the long run. Regarding regional stratification, domestic export sophistication in the eastern and western regions has more significant effects on promoting industrial upgrading than in the central region. In particular, in western regions, every increase in export sophistication by one unit will bring a significant industrial upgrading effect. Given this, China's new energy vehicles should increase export sophistication to help the country's industrial upgrading.

## 1. Introduction

For a long time, fossil energy has supported the development of industrial civilization but also brought environmental pollution, climate change, and other practical problems affecting human survival and growth; energy and environmental issues have become important in recent years. Energy production and consumption patterns based on fossil energy urgently need to be changed [1]. At the same time, the new energy industry is growing rapidly, and the world's wind, solar, and other clean energy power generation are in an accelerated development stage. There are still significant challenges in technological innovation, equipment development, engineering application, system security, and economy. All countries have pushed the development of new energy to an unprecedented height. Carbon dioxide is the gas produced during the petroleum, paraffin, coal, and natural gas combustion processes [2]. A significant increase in the supply of carbon dioxide in the atmosphere will gradually raise the Earth's surface temperature, resulting in global warming and a slew of unusual climate concerns. An essential source of carbon dioxide is motor vehicles [3]. The amount of carbon dioxide emitted is directly proportional to the amount of gasoline consumed by automobiles [4]. According to the data, the total exhaust emission from consuming 1 L of gasoline is approximately 2.5 kg, but the single component of carbon dioxide exceeds 2.3 kg [5]. Many countries and regions have issued various supportive policies to promote technological upgrading and market promotion of new energy vehicles. All countries' attitudes are relatively unified in supporting the development of new energy vehicles. After a period of development and life infiltration, because new energy vehicles have low power prices, environmental protection, and other advantages, they have gradually become an important choice for consumers to buy new energy vehicles. The development planning of new energy vehicles is divided into two categories: the timetable for banning the sale of fuel vehicles and the development goals of new energy vehicles [6].

The article "An Empirical Study on the Relationship between New Energy Vehicle' Export Sophistication and Industrial Structure Upgrading in China" was retracted in 2023. Reasons: signs of a paper mill; compromised peer review; unreliable results or conclusions.

The China Forum of Environment Journalists reported that global carbon dioxide emissions nearly reached 34 billion tonnes, with motor vehicles accounting for roughly 10% to 15% of total emissions in 2020. The Chinese Ministry of Transport reported that China's transportation sector emitted 820 million tonnes of greenhouse gas carbon dioxide in 2014, and road transport accounted for 690 million tonnes, approximately 84% of overall transport carbon dioxide emissions. It is a major source of carbon dioxide emissions. As a result, to minimize carbon dioxide emissions, motor vehicles and transportation will play a key role in replacing oil consumption with new energy on a broad scale, a method that is also the most direct and effective [7].

New energy vehicles include four types of hybrid electric vehicles (HEVs), battery electric vehicles (BEVs, including solar cars), fuel cell electric vehicles (FCEVs), and plug-in hybrids electric vehicles (PHEVs) expanding on the concept of the standard hybrid vehicle. They have both an internal combustion engine and a battery-powered electric motor. Nonconventional vehicle fuels refer to fuels other than gasoline and diesel [8]. The advancement of new energy vehicles involves many industries with long industrial chains and supply chains critical to national economic and social development [9]. Despite the impact of the COVID-19 pandemic, global energy vehicle stock growth grew rapidly from 2010 to 2020, with energy vehicle registration exceeding 10 million in 2020, a nearly 43% increase over 2019 [10]. China had 4.5 million new energy vehicles stock in 2020, accounting for 45% of the world's new energy vehicles, which is the world's largest trading country for new energy vehicles [11]. However, different categories of new energy vehicles in China are also confronted with the issue of technological growth mode [12]. If China vigorously promotes energy vehicle trade policies that ‘focus on quantity, not quality', the development of China's international auto industry's trade will almost certainly fall into the comparative advantage trap [13]. In fact, the market share of new energy vehicles in China has always been the largest in the low-end market represented by A00 models [14]. However, in recent years, according to the Passenger Association data, the proportion of A00 models had steadily decreased from 54.4% in 2017 to 15.0% in 2020, while the proportion of B-class vehicles has steadily increased from 4.3% in 2017 to 27.3% in 2020. This demonstrates that China's new energy vehicles are gradually progressing toward high-end and large-scale development markets [15].

The article "An Empirical Study on the Relationship between New Energy Vehicle' Export Sophistication and Industrial Structure Upgrading in China" was retracted in 2023. Reasons: signs of a paper mill; compromised peer review; unreliable results or conclusions.

As a result, China's cumulative sales of new energy vehicles have ranked first worldwide for seven consecutive years since 2015; improving the export sophistication of new energy vehicles trade is significant for promoting the upgrading of China's industry and realizing the transformation of China's foreign trade growth model [16]. Unfortunately, this topic has piqued the curiosity of only a few scholars thus far. Previous researchers only focused on new energy vehicle development and technological manufacturing but ignored the relationship between new energy vehicles and industrial upgrading. There has been little theoretical and empirical research on the relationship between the export sophistication of new energy vehicles and industrial upgrading in China [17]. As a unique growth point in China's economy after the production of fuel vehicles, developing new energy vehicles will bring new influences to China's industrial upgrading.

Based on this, the paper proposes relevant assumptions based on theoretical analysis and attempts to exploit China's 31 provinces, municipalities, and autonomous regions under the panel data to calculate China's export specialization of new energy vehicles and then introduces the index model with quantitative analysis on industrial upgrading and verifies theoretical assumptions [18]. Considering the unbalanced economic development in eastern, central, and western China, the heterogeneity of these three regions is further tested. A comprehensive analysis of the possible relationship between the domestic export sophistication of China's energy vehicle trade and industrial upgrading is done.

The article "An Empirical Study on the Relationship between New Energy Vehicle' Export Sophistication and Industrial Structure Upgrading in China" was retracted in 2023. Reasons: signs of a paper mill; compromised peer review; unreliable results or conclusions.

## 2. Literature Review

### 2.1. Industrial Upgrading

Industrial upgrading is defined as “the process by which economic actors, nations, firms, and workers move from low-value to relatively high-value activities in global production networks” [19]. The government and the market are the two main driving forces behind industrial upgrading. The first type involves the government backing leading industries and is the primary driver of industrial upgrading [20]. The second type is founded on comparative advantage, with industrial upgrading primarily depending on market power mechanisms. Concerning comparative advantage investment theory, comparative advantage is applied to international direct investment. With regard to dynamic comparative advantage investment theory, the theory of international direct investment illustrates how developing countries promote economic transformation through outward investment when economic development reaches a particular stage. FDI contributes to economic growth only when a sufficient absorptive capability of advanced technologies is available in the host economy. Economic development should align with the fundamental structure of capital and labour [21]. It must adhere to the economy's competitive advantage to accomplish long-term accumulation and constant upgrading of the industrial design to create sustainable economic growth. GDP is the overall reflection of the macroeconomic, covering all industries of the national economy, as well as all kinds of industrial economies; that is, the added value of the industrial economy is a part of GDP. Industrial upgrading and GDP growth are connected but distinct, with the development of industrial structure and quality representing an increase in production efficiency [22]. Although partial and gradual industrial upgrading may not improve a country's overall production efficiency and economic growth, comprehensive and radical industrial upgrading of leading companies is integrated with economic growth [23]. It inevitably enhances a country's overall production efficiency and economic development. The main element affecting a country's industrial upgrading and economic growth is technological advancement. Technological innovation helps developed countries advance technologically and upgrade their industrial structures. Mazzucato researched the United States as a high-income country's forefront of industrial technology worldwide. Therefore, if the United States wants to develop technologies and industries, it must rely on its research and development. America's economic success results from public and state-funded innovation and technology investments. R&D innovation is an essential channel for importing trade liberalization and improving manufacturing technological exports [24]. By contrast, developing countries mainly achieve technological progress and industrial structure upgrading through capital technology and imitation. As a result, from a trade perspective, industrial upgrading is primarily based on the ‘technology spillover' impact as defined by international trade theory [25]. The early achievements mainly explained the importance of a country participating in the division of labour from the perspective of factor endowment theory. Then, some scholars expounded on the benefits of participating in processing trade; export could promote industrial upgrading, and foreign trade should effectively drive industrial upgrading [26].

The article "An Empirical Study on the Relationship between New Energy Vehicle' Export Sophistication and Industrial Structure Upgrading in China" was retracted in 2023. Reasons: signs of a paper mill; compromised peer review; unreliable results or conclusions.

In fact, some scholars have long proposed that international trade does not lead to a country's industrial upgrading, and such developing countries may fall into the ‘international trade trap', where they become stuck in low-level and low-technology primary product processing for an extended period. Although there is no consensus on whether international trade would support industrial upgrading, these studies are essential for a thorough knowledge of international trade's influence on a country's or region's economic growth.

### 2.2. Automobile Industry

In industrialized nations, the development of the automobile industry is directly correlated with the development of the national economy and follows the same growth trajectory as GDP [27]. The added value of the automobile industry, on the other hand, indicates the ultimate outcomes of the industrial production operations of automobile industry firms in the form of money over a certain period. Since the gross domestic product (production method) is the sum of the added values of various departments, the proportion of the added value of the automobile industry in the gross domestic product reflects the impact of the automobile industry on the national economy.

According to China's data from 2004 to 2019, as can be shown in Figures 1 and 2, the automobile industry's added value in GDP (excluding the industrial chain) fell between 1.2% and 1.7%. The automobile industry's influence on the national economy is stable but growing, and the proportion of the automobile industry in manufacturing is increasing year by year. The contribution rate of China's automobile sector to GDP growth in 2019 was 0.36%, implying that the automobile industry generated 0.36% of the GDP growth rate in 2019.

The article "An Empirical Study on the Relationship between New Energy Vehicle' Export Sophistication and Industrial Structure Upgrading in China" was retracted in 2023. Reasons: signs of a paper mill; compromised peer review; unreliable results or conclusions.

The automobile industry not only leads to an expansion, which has repercussions across the economy, but also supports a comprehensive supply chain and generates a variety of commercial services [28]. International Energy Agency reports vehicle manufacturing is a strategic industry in Europe, where 18.5 million cars, vans, trucks, and buses are manufactured per year, and the turnover generated by the automotive sector represents 7% of Europe's total GDP in 2020. Automobile manufacturers operate approximately 226 vehicle assembly and production plants in Europe, generating government revenue that accounts for €440.4 billion in taxes in major European markets. The growth of the automobile industry has propelled the development of over 150 associated sectors, such as steel, machinery, electronics, rubber, glass, the chemical industry, construction, and services, and it could also boost the service industry. The European auto industry exports globally delivering quality ‘Made in Europe' products worldwide and generates a 74 billion trade surplus for Europeans. This international business could create skilled jobs; 14.6 million Europeans work in the auto industry (directly and indirectly), accounting for 6.7% of all European jobs. As the automotive industry accelerates its in-depth transformation to electrification, intelligence, interconnection, and sharing, the industrial categories covered by the industrial chain of new energy vehicles will continue to expand into new parts categories based on the original mechanical parts, structural parts, and electrical parts, such as batteries, motors, and ADAS systems. The automobile industry's added value share has increased as the industrial chain has continued to expand. This tendency will continue with the prospect of more significant development due to technical innovation and industrial improvement [29].

### 2.3. Export Sophistication

After the beginning of the millennium, the focus of academic study regarding international commerce switched from volume to technological substance and the productivity of trade commodities. The idea of industrial export sophistication represents a suitable research method for this shift, leading to a significant number of exploratory studies on export and import commerce in recent years from the perspective of export sophistication.

Export sophistication was first in the form of the trade sophistication index [30]. The index is based on the assumption that an export product is related to the income level of the country in which the product is exported. This is the earliest research on the measurement of export sophistication methodology, and many researchers have improved the index based on this. Hausmann et al.'s [31] research played a pioneering role in this field. He first proposed the concept of ‘export sophistication'. Countries with high-tech advantages export products with relatively high technology content, while labor-intensive countries export products with low-technology content. Lall extends the concept of complexity to international commerce and exports. Rodrik [32] expands on Hausmann's research by stating that the sophistication of a country's export technology, to some extent, reflects the position of a country's industry in the international division of labor [33]; that is, export sophistication can reflect the proportion of a country's exports of high-value and high-quality goods in all exports. The greater the share of such commodities in a country's exports, the higher the country's rank in the international division of labor and the greater the export sophistication of exports [34]. Following that, Hausmann et al. conducted a more in-depth investigation into the concept, stating that in such an international trade pattern, export sophistication is a comprehensive expression of a country's export commodities, including product value, technical content, and production efficiency, and it is a broad concept for export commodities research.

The article "An Empirical Study on the Relationship between New Energy Vehicle' Export Sophistication and Industrial Structure Upgrading in China" was retracted in 2023. Reasons: signs of a paper mill; compromised peer review; unreliable results or conclusions.

With the advancement of the world economy and new problems and trends in international trade, the concept of export sophistication has been put forward as a research focus in the field, providing a new perspective and research methods for the world division of labor pattern, transfer of international industry chain, emerging economies export structure optimization, and offering a novel method to improve global competitiveness.

In academic circles, there are now two mainstream measuring methods: one is based on Rodrik and Hausmann's EXPY index of per capita income, while the other is based on Schott's Export similarity index (ESI). EXPY assumes that the export sophistication of an overseas product is positively correlated with the exporting country's per capita income level, so the product's export sophistication is equal to the weighted average of all exporting countries per capita income, where the weight is the proportion of the total amount of the product's export in the world total of the product's export. The weighted average of the export sophistication of all the nation's export goods is the export sophistication of a country, and the weight is the proportion of the product's export in the country's overall export. The export simplicity index (ESI) assesses the degree to which a country's export commodity set and those of industrialized nations are comparable. The term ‘developed countries' refers to countries that are members of the OECD. The higher the export sophistication of a country's export, the more comparable its export structure is to OECD countries. The EXPY income index is more commonly used in industry and regional studies, and the ESI index is most widely used in cross-country studies. Chinese scholars estimate the complexity of China's export technology based on the above two methods but generally adopt Rodrik and Hausmann's per capita income EXPY index.

The article "An Empirical Study on the Relationship between New Energy Vehicle' Export Sophistication and Industrial Structure Upgrading in China" was retracted in 2023. Reasons: signs of a paper mill; compromised peer review; unreliable results or conclusions.

### 2.4. Influence of Export Sophistication on Industrial Upgrading

The Organization for Economic Cooperation and Development (OECD) divides the manufacturing industry into high-end technology, mid-high-end technology, mid-end technology, and low-end technology according to the different technological levels contained in the manufacturing industry. The industrial upgrading structure of the manufacturing industry is a process of transferring from low-end manufacturing to mid-end, mid-high-end, and then high-end manufacturing [35].

From the perspective of the relationship between the influence of regional and industry heterogeneity, many scholars confirm that the improvement of manufacturing technology complexity has a positive role in promoting the upgrading of the manufacturing industrial structure. In addition, there are regional and industrial differences in the effects of technological complexity improvement on industrial structure upgrading [36]. Varum et al. [37] studied the relationship between technological innovation and industrial structure optimization in the Portuguese manufacturing industry. The research results showed that technological innovation in the middle and high-end manufacturing industries could achieve high labor productivity, conducive to promoting the optimization of the country's industrial structure. Lin et al. [38] explored the promoting effect of human capital and technological progress on the structural optimization of the manufacturing industry based on China's provincial panel data from 2003 to 2017 and found that both played a significant role in promoting the structural optimization of the manufacturing industry, and the promoting effect had noticeable regional differences.

The theoretical analysis from the internal mechanism and the existing literature has also discussed the fundamental mechanism of industrial and technological complexity promoting industrial structure upgrading. According to Ngai and Pissarides [39], the relative changes in total factor productivity (TFP) between industries will form differences in the development of industries, and the relative increase of the share of enterprises with a higher TFP growth rate is the motivation for industrial structure upgrading.

The article "An Empirical Study on the Relationship between New Energy Vehicle' Export Sophistication and Industrial Structure Upgrading in China" was retracted in 2023. Reasons: signs of a paper mill; compromised peer review; unreliable results or conclusions.

Existing research on the association between technological complexity and industrial upgrading is mainly based on international panel data for horizontal comparison or using the national level of a country's time series data for the overall study. Not much research has been done on different sections of the country.

Hence, in this study, it is possible to assume that improving the export sophistication of China's new energy vehicles could upgrade China's transformation of foreign trade mode and enhance the upgrading of China's industry. Therefore, the following hypothesis is proposed:

  H1: developed regions have a higher export sophistication than less developed areas.
  H2: domestic export sophistication of the new energy vehicles industry has a significant positive stimulus effect on the industrial upgrading of China.
  H3: export sophistication as the internal influencing factor is important in the industrial upgrading of export trade structure. The external influencing factors are R&D, FDI, market, and per capita GDP growth rate which have less impact than internal influences.
  H4: the export sophistication of new energy vehicles in different regions has different effects on China's industrial upgrading.

## 3. Methodology and Data

### 3.1. Methodology

#### 3.1.1. Test the Export Sophistication

According to current theoretical research, the new energy vehicles trade export specialization index has a significant advantage in measuring the international competitiveness of a country's new energy vehicles export. It can be used as an auxiliary indicator to evaluate industrial upgrading. This methodology is based on Rodrik's and Hausmann's per capita income EXPY index calculation approach, which splits the technical process of export sophistication index of new energy vehicles trade into two parts.

However, the transfer of international industry makes developing countries process trade vigorously and become the center of the global manufacturing industry [40]. In this context, the technical content of export products in countries like China, which are mainly based on processing trade, is not all domestic technical contribution, which cannot reflect the country's technical level and industrial structure and will overestimate the actual technical level of export products. Therefore, when the EXPY model measures export technology complexity, it generally counts the value of a country's export products as its contribution, leading to an inaccurate interpretation of reality.

Scholars believe that the domestic input and intermediate input of export commodities should be distinguished [41], and the impact of processing trade on the calculation of export technology complexity should be excluded [42].

The article "An Empirical Study on the Relationship between New Energy Vehicle' Export Sophistication and Industrial Structure Upgrading in China" was retracted in 2023. Reasons: signs of a paper mill; compromised peer review; unreliable results or conclusions.

First, the index called PRODY is measured. This index is a weighted average of the per capita GDP of countries exporting a given product and thus represents the income level associated with that product, where province is indexed by *j*, and products are indexed by *k*. Total exports of province *j* are as follows:

(1) $$\begin{array}{c} X_{j}=\sum j\;x_{jk}. \end{array}$$

Let the per capita GDP of province *j* be denoted by *Y*_*j*_. Then, the productivity level is associated with product *k*; PRODY_*k*_ is as follows:

(2) $$\begin{array}{c} {\text{PRODY}}_{k}=\Sigma_{j}Y_{j}, \end{array}$$

where PRODY_*k*_ is an indicator that measures the relative competitive advantage of each product sector in the export trade of new energy vehicles, representing the export revenue value of each product. *X*_*jk*_ represents the export value of each product *k* in province *j*, *X*_*j*_ represents the entire export value of energy vehicle commerce of province *j*, *Y*_*j*_ represents the per capita income level of province *j*, and the per capita GDP of province *i* is denoted by *Y*_*j*_.

Second, the export sophistication EXPY_id_ of every province is measured. The formula is

(3) $$\begin{array}{c} {\text{EXPY}}_{jd}=\sum \alpha_{ij}{\text{PRODY}}_{i}+\left(1-\sum \alpha_{ij}\right){\text{PRODY}}_{j}, \end{array}$$

where *i* means intermediate products; ∑*α*_*ij*_ PRODY_*i*_ presents intermediate products' EXPY; *j* means final products *k*; (1−∑*α*_*ij*_) PRODY_*j*_ presents the value of the input in the domestic production process after the intermediate input technical complexity is removed, which represents the contribution of the production (assembly) process of the final product to its value, that is, the proportion of the value created by this process to the total value of the product 4. *α*_*ij*_ means input coefficient, reflecting the proportion of input to the final product; “Input coefficients” represent the scale of raw materials and fuels used can be obtained by dividing the input of raw materials and fuels utilized to generate one unit of production in each sector. EXPY_id_ means really domestic input value after deleting the intermediate products *i*.

#### 3.1.2. Empirical Analysis

We centralize variables of EXPY and industry upgrading to measure the effect. According to the Pey-Clark theory of industrial organization, industrial structure rational (ISR) is generally used to represent the adjustment of industrial structure. This study also uses this index to measure the change in China's industrial structure. Our model regression equation is specified as follows:

(4) $$\begin{array}{c} {\text{UP}}_{j,t}={\text{EXPY}}_{j,t}+\text{GDP}{\text{growth}}_{j,t}+\text{ R}\&{\text{D}}_{j,t}{+\text{ FDI}}_{j,t}+{\text{Market}}_{j,t}+{\text{R\&Dhr}}_{j,t}+\;\varepsilon_{j,t}. \end{array}$$

In the equation, UP_*j*,*t*_ denotes the dependent variable (index of China's industrial upgrading) and is measured by the ratio of the sum of secondary industry plus tertiary industry to GDP [43]. GDP growth_*j*,*t*_ denotes the growth rate of per capita GDP of each province [44, 45]. R&D_*i*,*t*_ presents provincial Research and development fund expenditure [17]. FDI_*j*,*t*_ is a foreign direct investment in one province [46]. To eliminate possible endogeneity issues, Market_*j*,*t*_ denotes the number of patents [47]. R&D hr_*j*,*t*_ represents the R&D human resources [48]. *i*, *t* is the error term. All data, except per capitaGDP growth rates, require logarithmic processing.

The article "An Empirical Study on the Relationship between New Energy Vehicle' Export Sophistication and Industrial Structure Upgrading in China" was retracted in 2023. Reasons: signs of a paper mill; compromised peer review; unreliable results or conclusions.

### 3.2. Data

This study covers the period 2010–2020 panel data and uses Stata 16.0. Data on China's new energy vehicles market are derived from the Customs Statistics China database. International business data on new energy vehicles are reported by UN COMTRADE, OECD, and WTO [49]. This paper selected and heterogeneous Figure 3 China's three major economic belts partition (‘Seventh Five-Year Plan of China in 1985–1990'): the eastern economic region (industrial region), the central economic region (hinterland regions), and the eastern economic region (backward region) [50, 51].

Based on an in-depth study of the HS code and the China Import and Export Tariff, this study revised the Harmonization System Code 6 (HS-Code 6), and the detailed categories of new energy vehicles and their HS 6 codes are shown in Table 1.

## 4. Empirical Analysis and Results

As can be seen from Figure 4, even though all three regions increase in these years, the eastern economic region (developed areas) in terms of high technology, high capital, and R&D human resources still has a strong technical advantage over less developed areas of China. The export sophistication of new energy vehicles in the eastern part of China with economically developed areas is higher than in the central regions and western regions in terms of export sophistication of new energy vehicles. As a result, hypothesis 1 has been put to the test.

Stationarity is the basic requirement for constructing the panel data regression model, so the IPS method is first used to test the stationarity of each variable (Table 2). As can be seen from the test results, at the 1% level, UP, R&D, FDI, GDP growth, R&D hr, EXPY, and Market belong to the first difference stability.

The article "An Empirical Study on the Relationship between New Energy Vehicle' Export Sophistication and Industrial Structure Upgrading in China" was retracted in 2023. Reasons: signs of a paper mill; compromised peer review; unreliable results or conclusions.

If there is a cointegration relationship between nonstationary sequences, it indicates that these variables directly have a long-term stable relationship with each other, which can also be used to build regression models. In this paper, the Pedroni test is used to test the cointegration of the data in this panel.  Table 3 shows that all cointegration test statistics passed the test at the 1% significance level, and it is considered that there is a long-term cointegration relationship between variables. Therefore, the panel data in this paper can be used to build a panel data regression model.

It shows the process of constantly introducing variables for regression. The effect coefficient in Table 4 means export sophistication on industrial upgrading is 1.11% at the highest level and 0.57% at the lowest level, implying that each percentage point increase in export sophistication of energy vehicles contributes 0.01% to industrial upgrading. Hypothesis 2 has therefore been proven true.

Although the coefficients of research and development variables, R&D, FDI, and market variables are all positive, the effect of these control variables on industrial upgrading is much smaller than the effect of the export sophistication index. Even though GDP growth and R&D hr variables have negative effects on industrial upgrading, hypothesis 3 has therefore been proven true.

Consider that in actual economic operations, the level of industrial upgrading at the outset has a considerable impact on the present position of industrial upgrading. Industrial upgrading is a dynamic process that occurs over time. As a result, it is crucial to incorporate industrial transformation indications and upgrade the explained variables throughout the lag period. This will result in many issues, including model endogeneity. Therefore, this chapter builds a dynamic panel model for regression analysis using 2SLS model estimates, and the regression findings are as follows. The results show that in Table 5, first L.EXPY was a significant and valid instrumental variable. Moreover, L2 EXPY was significant and positive. These results suggest considerate endogenous, and EXPY has a significant and positive promoting effect on industrial upgrading.

Due to the unbalanced development level of the three economic regions in China, this paper tests the regional heterogeneity of the relationship between EXPY and industrial grading.  Table 6 results revealed that in the three economic zones, only Eastern EXPY and Western EXPY are positive and significant, and the coefficient is not zero. This suggests that for every 1% increase in EXPY in the eastern and western regions, the industrial upgrading of their provinces will be completed by 0.5% and 0.8%. Although we can get that hypothesis 4 of EXPY on industrial upgrading is established in central and western China, the influence of EXPY in the western region is greater than that in the eastern region. In fact, according to the linear correlation results, China's EXPY has an impact on industrial upgrading, but the impact in central China on industrial upgrading is not the same as in eastern, central, and western China. Moreover, this result is in line with China's policies. At present, China attaches great importance to the development of western and eastern regions.

The article "An Empirical Study on the Relationship between New Energy Vehicle' Export Sophistication and Industrial Structure Upgrading in China" was retracted in 2023. Reasons: signs of a paper mill; compromised peer review; unreliable results or conclusions.

## 5. Conclusion

Industrial upgrading is unavoidable if countries are to reach a certain level of economic growth. Moreover, technical competitiveness has become essential in determining a country's international competitiveness. Hence, what is the connection between industrial upgrading and technological competitiveness? This paper is based on relevant academic research around the world, focusing on China's 31 provinces panel data from 2010 to 2020, which is divided into three economic regions: the eastern economic region (developed region), the central economic region (hinterlands region), and the eastern economic region (undeveloped region) to measure the export sophistication of new energy vehicles and especially observe the long-term and short-term effects to industry upgrading. Regression analysis was used to determine the factors influencing industry upgrading with China's export sophistication of new energy vehicles. The main conclusions are as follows.

Developed regions have advantages over undeveloped regions; improving the export sophistication index is conducive to realizing China's industrial upgrading.

In terms of China's new energy vehicles' export sophistication, there is a significant positive correlation between export sophistication and industrial upgrading. China's new energy vehicles industry is positively affected by EXPY, R&D, FDI, average GDP growth rate, and market factors, except R&D human recourse. But the economic development is a long-term process of dynamic change and development. The implementation of policies takes a certain period to have an effect. The short-term impact cannot impress whether long-term development is effective. In this study, in the process of a country or region's industrial upgrading, all factors will positively influence industrial upgrading from the standpoint of dynamic change range. First-order lag and second-order lag are still significant and stable, meaning that export sophistication could also promote industrial upgrading for a long time.

Due to the unbalanced development level of the three economic regions in China, this paper's heterogeneity tests the regional between export sophistication and industrial grading. This shows that for every 1% increase in export sophistication in the eastern and western regions, the industrial upgrading of their provinces will be completed by 0.5% and 0.8%. Although we can get the hypothesis of export sophistication on industrial upgrading established in China, in fact, according to the linear correlation, China's export sophistication has an impact on industrial upgrading. Still, the effect of central China on industrial upgrading is not the same as in eastern and western China. In terms of regional stratification, the export sophistication in the eastern and western regions has more significant effects on promoting industrial upgrading than in the central region in China. In particular, in western China, the current level of technology is still relatively low, and every increase in export sophistication by one unit will bring a significant industrial upgrading effect.

The article "An Empirical Study on the Relationship between New Energy Vehicle' Export Sophistication and Industrial Structure Upgrading in China" was retracted in 2023. Reasons: signs of a paper mill; compromised peer review; unreliable results or conclusions.

To develop the energy vehicle industry, promoting the export sophistication of new energy vehicles to complete industrial upgrading in China, the next stage could start from the following aspects.

First, governments should improve the ability of independent innovation and increase science and technology investment. Innovation factors have a significant positive effect on the overall improvement of China's new energy vehicles industry. Therefore, independent innovation ability is the core factor in promoting the progress of export sophistication in China's high-tech industry. Relying on learning and imitating the innovation of enterprises in other countries is not a long-term plan, nor can the core technology be mastered. Society could improve the innovation incentive range and encourage a national innovation atmosphere by increasing investment in technological innovation from the aspects of ideology and cultural environment.

Second, researchers should pay attention to sharing innovation resources. It can be seen from the empirical analysis that, although there are some different effects of various factors on the high-tech industries' export sophistication, there are also some commonalities in different regions of China. For example, FDI and R&D have specific positive effects on the export sophistication of the new energy vehicles industry at the national level and in the three economic regions; therefore, to maximize the overall export sophistication of China's new energy vehicles industry, enough attention should be paid to the mobility of innovation resources and innovation factors among different regions. In particular, we should encourage and advocate for provinces that are rich in innovation resources in eastern China to communicate with central and western provinces in China. Sharing innovation resources, innovation factors, and technical information improves the innovation spillover effect of high-tech industries in eastern areas and drives the increase of export sophistication of high-tech sectors in other regions and the whole of China.

The article "An Empirical Study on the Relationship between New Energy Vehicle' Export Sophistication and Industrial Structure Upgrading in China" was retracted in 2023. Reasons: signs of a paper mill; compromised peer review; unreliable results or conclusions.

Third, it is worth noting that although the coefficient of average GDP growth rate was positive after the model analysis, this shows that average GDP growth could not realize the goal of industrial upgrading. However, in a natural process of economic development, if GDP growth in terms of quantity is pursued while ignoring the improvement of ‘quality', then GDP growth not only brings disadvantages to the realization of the goal of industrial upgrading but also has a negative hindering effect under some conditions. In other words, in developing technology and economy in a country or region, successfully realizing society's economic growth by blindly pursuing GDP growth is not the most direct and effective policy tendency. A series of supporting measures, such as introducing and implementing policies on science, technology, education, and human capital cultivation, is necessary for the whole country.

Lastly, investment in educational research and development should be emphasized, because innovation is inextricably linked to talent, and talent cultivation is linked to education. Increasing education investment is another critical step in promoting the export sophistication of China's new energy vehicles and other high-tech industries. While popularizing education for all, the government should continue to invest in developing cutting-edge technical and professional abilities, providing a human capital foundation for China's ability to innovate independently.

## Figures and Tables

**Figure 1:** Contribution value of China's automobile industry to GDP for 2004–2019.

**Figure 2:** Contribution rates of China's automobile industry to GDP for 2004–2019.

**Figure 3:** China's three major economic belts partition.

**Figure 4:** Domestic EXPY results in three economic regions, 2010–2020.

**Table 1:** The categories of new energy vehicles and their key parts products and their Harmonized Commodity Description and Coding System (HS) codes.

HS 6	Commodity descriptions
870220	Compression ignition piston internal combustion engine (diesel or semidiesel engine) and the motor drive.
870230	Piston reciprocating combustion engine and drive the motor car.
870240	Passenger car with only the motor drive.
870340	Lighting reciprocating piston internal combustion engine and driving the motor car.
870350	Compression ignition piston internal combustion engine (diesel or semidiesel engine) and drive the motor car.
870360	Lighting reciprocating piston internal combustion engine and drive motor, can be plugged into external power supply for charging other manned vehicles.
870370	Compression ignition piston internal combustion engines (diesel or semidiesel engines) and other manned vehicles that drive motors, which can be recharged by plugging in an external power source.
870380	Other manned vehicles equipped with a drive motor only.
870911	Electrical tractors for short-distance transport of goods.
850650	Primary cells and primary batteries, lithium.
850760	Pure electric vehicle and plug-in hybrid vehicle, lithium-ion battery.

The article "An Empirical Study on the Relationship between New Energy Vehicle' Export Sophistication and Industrial Structure Upgrading in China" was retracted in 2023. Reasons: signs of a paper mill; compromised peer review; unreliable results or conclusions.

**Table 2:** Unit root test results.

Variables	Deterministic	Level	First difference
		ADF-Fisher	ADF-Fisher
UP	Intercept	100.7964^∗∗^(0.0013)	85.7072^∗∗^(0.0248)
	Intercept and trend	108.1052^∗∗∗^(0.0003)	81.5745^∗∗^(0.00485)

EXPY	Intercept	147.3221^∗∗∗^(0.0000)	135.8967^∗∗∗^(0.0000)
	Intercept and trend	133.3021^∗∗∗^(0.0000)	136.2904^∗∗∗^(0.0000)

R&D	Intercept	71.3696(0.1495)	80.8713^*∗*^(0.0375)
	Intercept and trend	85.4031^*∗*^(0.0173)	112.4023^∗∗∗^(0.0000)

Market	Intercept	53.6984(0.7038)	86.6596^∗∗^(0.0140)
	Intercept and trend	40.6731(0.9736)	182.3295^∗∗∗^(0.0000)

FDI	Intercept	124.5645^∗∗∗^(0.0000)	208.9380^∗∗∗^(0.0000)
	Intercept and trend	135.6121^∗∗∗^(0.0000)	125.7779^∗∗^(0.0000)

R&D hr	Intercept	103.9746^∗∗∗^(0.007)	161.6015^∗∗∗^(0.0000)
	Intercept and trend	92.8166^∗∗∗^(0.0068)	123.2135^∗∗∗^(0.0000)

GDP growth	Intercept	45.2668(0.9455)	405.8836^∗∗∗^(0.0000)
	Intercept and trend	40.0646(0.9863)	154.4162^∗∗∗^(0.0000)

Significance: ^∗∗∗^*p* < 0.01, ^∗∗^*p* < 0.05, and ^*∗*^*p* < 0.1.

**Table 3:** Cointegration tests results (Pedroni).

Variables	Statistic	*p* value
Modified Phillips-Perron *t*	6.8053	0.0000
Phillips-Perron *t*	−5.3917	0.0000
Augmented Dickey-Fuller *t*	−7.2758	0.0000

**Table 4:** Fixed effect analysis.

VAR	Model 1	Model 2	Model 3	Model 4	Model 5	Model 6
	UP	UP	UP	UP	UP	UP
EXPY	0.0111^∗∗∗^	0.0069^∗∗^	0.0061^∗∗^	0.0057^∗∗^	0.0058^∗∗^	0.0057^∗∗^
	(3.9327)	(2.4448)	(2.3552)	(2.1431)	(2.1563)	(2.1293)

R&D		0.0177^∗∗∗^	0.0152^∗∗∗^	0.0141^∗∗∗^	0.0156^∗∗^	0.0157^∗∗^
		(3.8580)	(2.8970)	(2.8141)	(2.7021)	(2.7368)

Market			0.0000	0.0000	0.0000	0.0000
			(1.1361)	(1.0918)	(0.9965)	(0.9807)

FDI				0.0004	0.0004	0.0004
			(1.0263)	(1.0277)	(1.0818)

R&Dhr					−0.0001	−0.0001
					(−0.8385)	(−0.8361)

GDP growth						0.0049
						(0.8458)

Constant	0.8236^∗∗∗^	0.8245^∗∗∗^	0.8314^∗∗∗^	0.8333^∗∗∗^	0.8323^∗∗∗^	0.8319^∗∗∗^
	(41.2261)	(43.3409)	(47.4539)	(47.9682)	(47.5014)	(46.7948)

Year FE	YES	YES	YES	YES	YES	YES
Province FE	YES	YES	YES	YES	YES	YES
Observations	316	316	316	316	316	316
*R*-squared	0.0931	0.2009	0.2107	0.2212	0.2239	0.2256
Number of id	31	31	31	31	31	31

Robust *t*-statistics in parentheses: ^∗∗∗^*p* < 0.01, ^∗∗^*p* < 0.05, and ^*∗*^*p* < 0.1.

The article "An Empirical Study on the Relationship between New Energy Vehicle' Export Sophistication and Industrial Structure Upgrading in China" was retracted in 2023. Reasons: signs of a paper mill; compromised peer review; unreliable results or conclusions.

**Table 5:** Autocorrelation 2SLS test.

	Model 1	Model 2	Model 3
	UP	UP	UP
EXPY	0.006^∗∗∗^	0.001	−0.001
	(0.002)	(0.002)	(0.002)

FDI	0.000^∗∗^	0.000	0.000
	(0.000)	(0.000)	(0.000)

GDP growth	0.005	−0.001	0.004
	(0.006)	(0.008)	(0.005)

R&D	0.016^∗∗∗^	0.010^∗∗^	0.005
	(0.004)	(0.004)	(0.004)

R&D hr	−0.000	0.000	0.000^*∗*^
	(0.000)	(0.000)	(0.000)

Market	0.000	0.000^*∗*^	0.000^∗∗^
	(0.000)	(0.000)	(0.000)

L.EXPY		0.005^∗∗^	
		(0.002)	

L2.EXPY			0.007^∗∗∗^
			(0.002)

_Cons	0.831^∗∗∗^	0.839^∗∗∗^	0.846^∗∗∗^
	(0.014)	(0.018)	(0.018)

*N*	307.000	270.000	239.000
*r * ^2^	0.234	0.207	0.215
*r * ^2^_a	0.135	0.085	0.075

^*∗*^ *p* < 0.1, ^∗∗^*p* < 0.05, and ^∗∗∗^*p* < 0.01.

**Table 6:** Heterogeneity results.

VAR	Eastern	Central	Western
	UP	UP	UP
EXPY	0.005^*∗*^	0.001	0.008^∗∗∗^
	(1.69)	(0.20)	(3.24)

FDI	0.000	0.000	−0.000
	(0.42)	(0.32)	(−0.44)

GDP growth	0.007	−0.010	0.003
	(1.30)	(−0.59)	(0.30)

R&D	0.002	0.003	0.018^∗∗∗^
	(0.69)	(0.22)	(2.98)

R&D hr	−0.000	0.004^∗∗∗^	−0.000^∗∗∗^
	(−0.73)	(3.34)	(−2.66)

Market	0.009^∗∗∗^	0.004	0.003^∗∗∗^
	(6.35)	(1.07)	(2.85)

_Cons	0.833^∗∗∗^	0.822^∗∗∗^	0.798^∗∗∗^
	(39.63)	(21.93)	(55.47)

*N*	113	87	107
*R * ^2^	0.485	0.387	0.391
Adj. *R*^2^	0.40	0.27	0.28

^*∗*^ *p* < 0.1, ^∗∗^*p* < 0.05, and ^∗∗∗^*p* < 0.01.

## Data Availability

All data, models, and code generated or used during the study are included in the submitted article.
